The article "Ginsenoside Rh4 Inhibits Colorectal Cancer Cell Proliferation by Inducing Ferroptosis via Autophagy Activation" was published in 2022. Journal: Evid Based Complement Alternat Med.

# Ginsenoside Rh4 Inhibits Colorectal Cancer Cell Proliferation by Inducing Ferroptosis via Autophagy Activation

**DOI:** 10.1155/2022/6177553

**Published:** 2022-05-29

**Authors:** Yingchao Wu, Dajin Pi, Yiliu Chen, Qian Zuo, Shuyao Zhou, Mingzi Ouyang

**Affiliations:** ^1^School of Traditional Chinese Medicine, Jinan University, Guangzhou, Guangdong 510632, China; ^2^MOE Key Laboratory of Tumor Molecular Biology and Key Laboratory of Functional Protein Research of Guangdong Higher Education Institutes, Institute of Life and Health Engineering, College of Life Science and Technology, Jinan University, Guangzhou, Guangdong 510632, China; ^3^College of Forestry and Landscape Architecture, South China Agricultural University, Guangzhou, Guangdong 510642, China

## Abstract

Colorectal cancer (CRC) is a severe threat to human health. Ginsenosides such as ginsenoside Rh4 have been widely studied in the antitumor field. Here, we investigated the antiproliferative activity and mechanism of Rh4 against CRC in vivo and in vitro. The CRC xenograft model showed that Rh4 inhibited xenograft tumor growth with few side effects (*p* < 0.05). As determined by MTT colorimetric assays, Western blotting, and immunohistochemical analysis, Rh4 effectively inhibited CRC cell proliferation through autophagy and ferroptosis (*p* < 0.05). Rh4 significantly upregulated autophagy and ferroptosis marker expression in CRC cells and xenograft tumor tissues in the present study (*p* < 0.05). Interestingly, the ferroptosis inhibitor ferrostatin-1 (Fer-1) reversed Rh4-induced ferroptosis (*p* < 0.05). Moreover, the autophagy inhibitor 3-methyladenine (3-MA) also reversed Rh4-induced ferroptosis (*p* < 0.05). These results indicate that Rh4-induced ferroptosis is regulated via the autophagy pathway. In addition, Rh4 increased reactive oxygen species (ROS) accumulation, leading to the activation of the ROS/p53 signaling pathway (*p* < 0.05). Transcriptome sequencing also confirmed this (*p* < 0.05). Moreover, the ROS scavenger N-acetyl-cysteine (NAC) reversed the inhibitory effect of Rh4 on CRC cells (*p* < 0.05). Therefore, this study proves that Rh4 inhibits cancer cell proliferation by activating the ROS/p53 signaling pathway and activating autophagy to induce ferroptosis, which provides necessary scientific evidence of the great anticancer potential of Rh4.

## 1. Introduction

According to the World Cancer Report, colorectal cancer (CRC) is one of the most dangerous malignant tumors in humans. CRC is the third leading cause of new cancer and the second leading cause of cancer death. The number of deaths in 2020 was 935,000 [1]. Surgery, radiotherapy, chemotherapy, and combination therapy are the primary treatment methods for CRC [2]. Although medical and surgical developments have extended the overall survival of patients, CRC still has a poor long-term prognosis, high recurrence rate, low five-year postoperative survival, and high tumor metastasis rate, which reduce therapeutic efficacy [3]. Despite the development of molecular targeted drugs with fewer side effects, chemotherapy is, in many cases, the most commonly used treatment for CRC patients. However, these chemotherapeutic agents can cause a range of dose-limiting toxicity (DLT) symptoms, such as weight loss and heart, liver, and kidney toxicity [4]. The critical challenge in cancer treatment is how to effectively kill cancer cells without affecting healthy cells. Therefore, finding effective antitumor drugs with few side effects is still necessary.

The use of traditional Chinese medicinal herbs with low toxicity as alternatives to antitumor drugs has attracted widespread attention [5]. In past clinical reports, traditional Chinese herbal medicines (*Panax ginseng*, *Panax notoginseng*, and American ginseng) have been widely used to treat malignant tumors and prevent and treat tumor-related adverse reactions [6–8]. Ginsenoside is the primary pharmacologically active component of ginseng and has a wide range of biological activities, including immunoregulatory [9], anti-inflammatory [10,11], antioxidative [12], neuroprotective [13], antidiabetic [14], antiobesity [15], and antileukemic [16] effects, in addition to its use in treating cardiovascular diseases [17] and its antitumor effects [18]. The types of ginsenoside compounds vary and include Rb1, Rb2, Rc, Rd, Re, Rf, Rg1, Rg2, Rg3, Rh1, Rh2, Rh3, and Rh4. The most common ginsenosides are Rb1, Rd, Re, Rg1, Rg3, and Rh1 [19]. In previous studies, some ginsenosides, such as Rg1, Rg2, Rg3, Rh2, Rh3, and Rh4, showed antitumor activity by inducing apoptosis and autophagy to suppress migration or inhibit proliferation [20–24]. Ginsenoside Rh4 (Rh4) is a rare triol ginsenoside that is characterized by being more soluble in water than other polysaccharide ginsenosides [25]. Good solubility can improve its clinical application prospects.

Ferroptosis is a novel type of regulated cell death caused by iron-dependent lipid peroxidation [26]. This form of cell death is characterized by increased levels of intracellular reactive oxygen species (ROS), iron, and lipid ROS concentrations and lacks the typical manifestations of apoptosis [27], necrosis [28], and pyroptosis [29]. Thus, this death process cannot be inhibited by apoptosis, necrosis, or pyroptosis inhibitors, but it can be inhibited by antioxidants and iron-chelating agents [30,31]. It has been reported that ginsenosides can increase ROS concentrations in cancer cells [32]. Furthermore, the main reason for tumor treatment resistance is that tumor cells often have defects in cell death mechanisms. Compared with normal noncancerous cells, cancer cells need high levels of iron to survive and grow. This iron dependence makes cancer cells more prone to iron-mediated cell death, also known as ferroptosis [33]. Therefore, ferroptosis induction may be a potential novel antitumor strategy for CRC.

Previous studies have shown that Rh4 has anticancer activity by inducing autophagic cell death via ROS/p53 signaling pathway in CRC cells [24]. During autophagy, cells form de novo structures called phagocytes, which elongate to engulf cytoplasmic proteins and even complete organelles in a double membrane structure named the autophagosome. Later, autophagosomes fuse with lysosomes, resulting in degradation of their contents [34]. Intriguingly, our recent study showed that Rh4 could induce ferroptosis in CRC cells. To date, there have been no reports of Rh4 inducing ferroptosis in CRC cells. However, the relationship between the Rh4-induced autophagy pathway and ferroptosis remains unclear. These years, p53 is found to be a master regulator of ferroptosis [35–37], and autophagy also plays an important role in ferroptosis [38]. Therefore, the purpose of this study was to explore the mechanism of Rh4-induced ferroptosis and whether the induction process was regulated by the autophagy pathway, which could significantly deepen our understanding of the use of Rh4 in CRC treatment. Finally, we showed the anti-CRC activity of Rh4 in vivo and in vitro. Our results show that Rh4 can induce autophagy and ferroptosis in CRC cells; moreover, the autophagy pathway regulates ferroptosis and is associated with increased ROS levels and p53 signaling pathway activation. Therefore, Rh4 can effectively inhibit the growth of CRC.

## 2. Methods and Materials

### 2.1. Rh4 Preparation

Rh4 (B24742, purity >98%) was purchased from Shanghai Yuanye Bio-Technology Co., Ltd. (Shanghai, China); dissolved in DMSO at a concentration of 100 mM for in vitro experiments; and dissolved in phosphate-buffered saline (PBS) at a concentration of 50 mg/mL for in vivo experiments. The Rh4 solution was stored at −80°C for later use.

### 2.2. Other Chemicals and Reagents

Dulbecco's modified Eagle's medium; high glucose; L-glutamine, phenol red (DMEM, 11965092); fetal bovine serum (FBS, 10270106); penicillin/streptomycin (10378016); PBS (10010023); trypsin-EDTA; 0.05% phenol red (25200072); and 3-(4,5-dimethylthiazol-2-y1)-2,5-diphenyltetrazolium bromide (MTT, V13154) were supplied by Gibco (NY, USA). Giemsa staining solution (C0133) was purchased from Beyotime Institute of Biotechnology (Shanghai, China). N-acetyl-cysteine (NAC, A9165), 3-methyladenine (3-MA, M9281), ferrostatin-1 (Fer-1, SML0583), Z-VAD-FMK (Z-VAD, V116), necrostatin-1 (Nec-1, N9037), and belnacasan (VX-765, 5313720001) were purchased from Sigma-Aldrich (Darmstadt, Germany). Primary antibodies against p53 (60283-2-Ig), p62 (66184-1-Ig), Beclin1 (11306-1-AP), xCT/SLC7A11 (26864-1-AP), and GPX4 (67763-1-Ig) were purchased from Proteintech (Wuhan, China). Primary antibodies against Atg7 (8558T), LC3A/B (12741S), KEAP1 (8047S), NRF2 (12721T), NCOA4 (66849S), FTH1 (4393S), DMT1/SLC11A2 (15083S), and GAPDH (5174S) and rabbit (7074P2) or mouse (7076P2) secondary antibodies were purchased from Cell Signaling Technology (Danvers, MA, USA). For in vitro experiments, Rh4 was dissolved in DMSO and medium, and the final concentration of DMSO in medium was ≤0.3% (vol/vol).

### 2.3. Cell Culture

The human CRC cell lines HT29, HCT116, DLD1, and RKO were gifts from the Life Science and Technology College, Jinan University (Guangzhou, China). The cells were cultured in DMEM supplemented with 10% FBS, 100 U/mL penicillin, and 100 *µ*g/mL streptomycin in a 5% CO_2_ incubator (Thermo Fisher Scientific, Waltham, MA, USA) at 37°C. The medium was changed every 72 hours, and the cells were routinely subcultured when the cells reached 90% confluence. Logarithmic growth phase CRC cells were used to conduct the experiments. If the experimental process needs to be treated with inhibitors, the use method is pretreatment for 4 hours.

### 2.4. Analysis of Cell Viability

Cell viability was measured by the MTT colorimetric assay. CRC cells were seeded in 96-well plates (8 × 10^3^, 5 × 10^3^, or 3 × 10^3^ cells/well in 100 *μ*L) and cultured for 12 hours. To determine different dose-dependent effects, the original medium was discarded, and 100 *μ*L of DMEM-diluted Rh4 solution was added to each well at final concentrations of 0, 25, 50, 100, 150, 200, and 300 *μ*M, or the cells were pretreated with different inhibitors before the addition of Rh4-containing medium. The cells were cultured with Rh4-containing medium for 24, 48, or 72 hours before the MTT colorimetric assay was performed. After culture, 20 *μ*L of MTT solution (5 mg/mL) was added to each well. After the cells were cultured for 4 hours at 37°C, the supernatant was discarded, and 150 *μ*L of DMSO was added to each well and stirred well for 15 minutes. The absorbance of each well was then measured with a microplate reader (BioTek Epoch, Vermont, USA) at a wavelength of 490 nm (A490). The recorded optical density (OD) values represented cell vitality. Then, the cell viability rate was calculated using the following equation: cell viability rate=(OD Sample/OD Control) × 100%. These experiments were performed in triplicate.

### 2.5. Assessment of Colony Formation

HT29 and HCT116 cells were seeded in 6-well plates (500 cells/well in 2000 *μ*L) and cultured for approximately 14 days. Colonies with more than 50 cells per colony were treated with 0.2% (vol/vol) DMSO or Rh4-containing medium (50, 100, and 200 *μ*M) for 48 hours. Subsequently, the medium was removed, and the cells were washed twice with PBS. After the cells were fixed with 4% paraformaldehyde, the colonies were stained with Giemsa stain for 5 minutes, and pictures were taken to record the results. These experiments were performed in triplicate, and ImageJ was used for quantitative analysis.

### 2.6. Assessment of Cell Growth

HT29 and HCT116 cells were seeded in 6-well plates (50,000 cells/well in 2000 *μ*L) and cultured for 12 hours. After 12 hours of culture, the original medium was discarded, and 2 mL of DMEM-diluted Rh4 solution was added to each well at a final concentration of 0, 50, 100, or 200 *μ*M. Two of the wells containing 200 *μ*M Rh4 were pretreated with 3-MA or Fer-1. After 48 hours of culture, the medium was discarded, fresh complete medium was added, and photographs were taken immediately under an inverted microscope at 100× magnification (Nikon, Japan).

### 2.7. Human CRC Xenograft Mouse Model

A total of 40 five-week-old BALB/c nude mice (15 ± 1 g) were purchased from Model Animal Research Center of Nanjing University (Nanjing, China). All experiments were conducted according to the relevant laws and institutional guidelines and with the approval (Approval No. IACUC-20201231-04) of the Animal Ethics Committee of Jinan University [SYXK (YUE) 2017–0174]. After acclimation for 10 days, the mice were randomly divided into two groups and inoculated with HT29 or HCT116 cells (1 × 10^7^ cells/100 *µ*L each) in the right forelimb pit. When the tumor grew to 100 mm^3^, mice in each group were randomly divided into two subgroups (*n* = 10): the control group (solvent) and the Rh4-treated group (i.p., 40 mg/kg/d). The body weights and tumor volumes were measured every 3 days, and the tumor size was calculated using the following equation: tumor volume = length × width^2^ × 1/2. Twenty-one days after treatment, the mice were anesthetized with pentobarbital (i.p., 150 mg/kg) and sacrificed by cervical dislocation. The xenograft tumor tissues, heart, liver, and kidneys were resected for subsequent experiments.

### 2.8. Hematoxylin and Eosin (HE) Staining

The fresh heart, liver, and kidney tissues were fixed with 4% paraformaldehyde, dehydrated, embedded in paraffin, cut into 5 *μ*m slices, then stained by hematoxylin for 30 min and eosin for 5 min, vitrified with xylene, and sealed with neutral resin. The stained slices were observed and photographed under a light microscope at 100× magnification (NIKON Eclipse Ci, Japan).

### 2.9. Western Blotting

Cells and xenograft tumor tissue samples were lysed in RIPA buffer (Beyotime Biotechnology, Shanghai, China) containing 1 mM phenylmethylsulfonyl fluoride (PMSF) (Beyotime Biotechnology, Shanghai, China) and 1× protease and phosphatase inhibitor cocktail (Beyotime Biotechnology, Shanghai, China) on ice. The lysates were then centrifuged at 12,000 *g* for 15 minutes at 4°C, and the protein concentration in the obtained supernatant was determined using an Enhanced BCA Protein Assay Kit (Beyotime Biotechnology, Shanghai, China). Equal amounts of protein were separated via SDS-PAGE and transferred to polyvinylidene fluoride (PVDF) membranes (Merck KGaA, Darmstadt, Germany). Next, the PVDF membranes were blocked with Tris-buffered saline plus Tween-20 (TBST) containing 5% skim milk for 1 hour and incubated with the indicated primary antibodies, including mouse anti-p53 (1 : 2000), anti-p62 (1 : 1000), rabbit anti-Beclin1 (1 : 1000), anti-Atg7 (1 : 1000), anti-LC3A/B (1 : 1000), anti-KEAP1 (1 : 1000), anti-NRF2 (1 : 1000), anti-NCOA4 (1 : 1000), anti-FTH1 (1 : 1000), anti-DMT1/SLC11A2 (1 : 1000), anti-xCT/SLC7A11 (1 : 1000), anti-GPX4 (1 : 1000), and anti-GAPDH (1 : 3000), after which the membranes were incubated with the corresponding secondary antibodies (1 : 5000). Finally, an ECL system (Bio-Rad Laboratories Inc., California, USA) was used to analyze the immune complexes. These experiments were performed in triplicate, and ImageJ was used for quantitative analysis.

### 2.10. Measurement of Intracellular and Xenograft Tumor Tissue ROS Concentrations

2′,7′-Dichlorodihydrofluorescein diacetate (DCFH-DA) staining (MAK143, Sigma, USA) was used to measure intracellular ROS concentrations. A tissue ROS assay kit (BB-470532, BestBio, Shanghai, China) was used to measure xenograft tumor tissue ROS concentrations. In short, after the cells were treated with different concentrations of Rh4 for 48 hours or fresh xenograft tumor tissues were collected, the ROS concentration in cells and xenograft tumor tissues was measured by flow cytometry (Agilent, California, USA) or a fluorescence microplate reader (BioTek, Vermont, USA), respectively, according to the kit instructions. These experiments were performed in triplicate. The data are expressed as the percentage of the fluorescence intensity relative to that of the control group.

### 2.11. Measurement of Intracellular and Xenograft Tumor Tissue GSH Concentrations

GSH and GSSG assay kits (S0053, Beyotime, Shanghai, China) were used to measure intracellular and tissue GSH concentrations. In brief, cells that were incubated in medium containing different concentrations of Rh4 for 48 hours or fresh xenograft tumor tissues were collected, and the experimental data were determined with a microplate reader according to the kit instructions. These experiments were performed in triplicate. The data are expressed in *μ*mol/mg.

### 2.12. Iron Assay

An iron assay kit (MAK025, Sigma, USA) was used to measure iron concentrations in cells or tissues. Cells were treated with different concentrations of Rh4 in medium for 48 hours (2 × 10^6^), or fresh xenograft tumor tissue (10 mg) was rapidly homogenized in 5 volumes of iron assay buffer. The samples were centrifuged at 16,000 *g* for 10 minutes at 4°C to remove insoluble material. The assay was performed according to the kit instructions. A microplate reader was used to measure the absorbance at 593 nm (A593). These experiments were performed in triplicate. The data are expressed in nmol/L.

### 2.13. Measurement of Intracellular Lipid ROS Concentrations

C11-BODIPY (D3861, Thermo, USA) was used to measure intracellular lipid ROS concentrations according to the manufacturer's instructions. Briefly, after being treated with different concentrations of Rh4 in medium for 48 hours, the cells were then cultured with 100 *μ*mol/L C11-BODIPY for 30 minutes at 37°C. The samples were washed twice with PBS. Then, the fluorescence intensities were measured at an emission wavelength of 510 nm and an excitation wavelength of 488 nm using a fluorescence microplate reader. These experiments were performed in triplicate. The data are expressed as the percentage of the fluorescence intensity relative to that of the control group.

### 2.14. Measurement of MDA Concentrations

A Lipid Peroxidation MDA Assay Kit (S0131S, Beyotime, Shanghai, China) was used to measure MDA concentrations in cells or tissues. In brief, cells were treated with different concentrations of Rh4 in medium for 48 hours or fresh xenograft tumor tissues were collected, and the experimental data were determined with a microplate reader according to the kit instructions. These experiments were performed in triplicate. The data are expressed in *μ*mol/mg.

### 2.15. Transcriptome Sequencing and Its Data Analysis

In consideration of financial problems and practical application scenarios of drugs, only HT29 xenograft tumor tissue samples were analyzed in this study. Transcriptome sequencing and data analysis of the samples were completed by Beijing Novogene Biotechnology Co., LTD. In short, there are two parts: sample collection and preparation and data analysis. The clustering and sequencing process is performed using the Illumina NovaSeq platform. Differential expression analysis of two groups (three biological replicates per group) was performed using the DESeq2 R package (1.20.0). Gene Ontology (GO) and Kyoto Encyclopedia of Genes and Genomes (KEGG) pathway enrichment analysis of differentially expressed genes were implemented by the clusterProfiler R package, in which gene length bias was corrected. An adjusted *P* value represents credibility of differences. The lower the *P* value, the higher the credibility. Original datasets for transcriptome sequencing can be obtained by accessing the NCBI Trace Archive or NCBI Sequence Read Archive (URL: https://www.ncbi.nlm.nih.gov/Traces/study/?acc=PRJNA826695).

### 2.16. Immunohistochemical Staining

Formalin-fixed xenograft tumor tissue samples were embedded in paraffin, and the paraffin-embedded samples were then cut into serial sections (4 mm thick). These sections were immunostained with the indicated primary antibodies, including anti-p53 (1 : 1600), anti-p62 (1 : 1000), anti-Beclin1 (1 : 100), anti-xCT/SLC7A11 (1 : 100), and anti-GPX4 (1 : 500), followed by incubation with the corresponding secondary antibodies (1 : 3000). Images were captured under a light microscope (Leica, Germany).

### 2.17. Statistical Analysis

The experimental data were analyzed using Student–Newman–Keuls (S-N-K) in ANOVA with SPSS version 13.0 software (SPSS Inc., IL, USA) or GraphPad Prism 9 (GraphPad Software, LLC, California, USA). The results are presented as the mean values ± standard deviation (SD). A *P* value < 0.05 was considered statistically significant.

## 3. Results

### 3.1. Ginsenoside Rh4 Can Inhibit CRC Cell Proliferation In Vitro and In Vivo

The chemical structural formula of Rh4 is shown in Figure 1(a). To evaluate whether Rh4 can inhibit CRC cell proliferation, we first established an in vitro model of CRC using HT29, HCT116, DLD1, and RKO cells. The MTT colorimetric assay revealed that Rh4 could significantly inhibit CRC cell proliferation. Rh4 dose-dependently and time-dependently inhibited the proliferation of four types of colon cancer cells compared with that in the control group (0 *μ*M Rh4, 0.3% DMSO or 24 hours) (Figures 1(b)–1(e)). The results showed that HT29 and HCT116 cells were more sensitive to Rh4, so we selected these two cells for subsequent experiments. For example, when cells were incubated in Rh4-containing medium for 48 hours, the inhibition rate induced by 200 *μ*M Rh4 reached 48.5 ± 1% in HT29 cells and 54.3 ± 0.9% in HCT116 cells. The IC50 values of Rh4 in inhibiting the proliferation of HT29 and HCT116 cells were 196.89 ± 1.71 *μ*M and 177.89 ± 2.45 *μ*M, respectively. In addition, the number of clones of HT29 and HCT116 cells was significantly decreased by Rh4 in a dose-dependent manner (Figures 1(f) and 1(g)).

Then, to verify whether Rh4 can inhibit growth in vivo, we inoculated HT29 or HCT116 cells into nude mice to establish a xenograft mouse model of CRC. The mice were injected with solvent or Rh4 (40 mg/kg/d). After 21 days of treatment, xenograft tumor size in the Rh4 group was significantly reduced compared with that in the control group, and the inhibition rates were 68.4% in HT29 cells and 70.3% in HCT116 cells (Figures 1(j)–1(l)). However, there was a significant difference in body weight between the control and Rh4 groups (Figure 1(h)). Body weight in the Rh4 treatment group (22.28 ± 0.30 g) was significantly higher than that in the solvent treatment group (20.54 ± 0.30 g). Meanwhile, HE staining showed that Rh4 had no significant damage to heart, liver, or kidneys (Figure 1(i)), suggesting that Rh4 has fewer toxic side effects. Therefore, these data suggest that Rh4 can significantly suppress CRC in vivo and in vitro without causing damage to organisms.

### 3.2. Ginsenoside Rh4 Can Activate Autophagy in CRC Cells In Vitro

To elucidate the functional role of Rh4 in inhibiting CRC, we used different pathway inhibitors to explore the effect of Rh4 on cell death. Rh4 significantly inhibited the growth of HT29 cells, and this effect was not reversed by inhibitors of apoptosis, necrosis, and pyroptosis. Moreover, the inhibitory effects on HT29 cell proliferation were reversed by ROS scavengers and autophagy and ferroptosis inhibitors (Figure 2(a)). Similar effects were observed in HCT116 cells, but apoptosis inhibitors also reversed the inhibitory effect of Rh4 on HCT116 cells (Figure 2(b)). The possible reason for this phenomenon is that HT29 cells have mutations at the p53R273H site, leading to loss of p53-mediated apoptosis [39], while Rh4 has been confirmed to induce apoptosis of HCT116 cells by activating p53 signaling pathway [24]. Interestingly, several drugs have been shown to enable mutated p53 to maintain normal autophagy regulation [40,41]. To verify that autophagy and ferroptosis inhibitors could reverse Rh4-mediated inhibition in HT29 and HCT116 cells, we used an inverted optical microscope and observed that the number of cells increased significantly after 48 hours of culture in 200 *μ*M Rh4 and pretreatment with autophagy or ferroptosis inhibitors (Figure 2(c)). During the experiment, we found an interesting phenomenon that HT29 cells grew in a stack, while HCT116 cells grew in a tiled pattern. Therefore, although MTT results showed a higher inhibition rate of Rh4 against HCT116 cells at the same concentration, assessment of colony formation (Figure 1(f)) and assessment of cell growth (Figure 2(c)) seemed to see a higher density of HCT116, which could also obtain the answer from the control group (0 *μ*M Rh4) between them (HT29 and HCT116) in Figures 1(f) and 2(c).

To verify whether Rh4 activates autophagy, we analyzed the protein expression level in cultured cells in vitro. Western blotting showed that Rh4 increased the expression level of the tumor suppressor gene protein p53 and the autophagy-associated protein LC3B in a dose-dependent manner. The expression levels of Beclin1 and Atg7, which are involved in autophagosome formation, also increased in a concentration-dependent manner, while p62 expression was significantly downregulated (Figures 2(d)–2(f)). To confirm whether the inhibition of Rh4-induced autophagy by autophagy inhibitors was reflected in the protein expression level, the autophagy inhibitor 3-MA was used prior to Rh4 treatment. Western blotting showed that the expression level of autophagy-related proteins in HT29 and HCT116 cells induced by 200 *μ*M Rh4 was significantly reversed by pretreatment with 3-MA, but the effect on p53 protein expression was not significant. Therefore, Rh4 can activate autophagy in CRC cells and promote cell death.

### 3.3. Ginsenoside Rh4 Can Induce Ferroptosis in CRC Cells In Vitro

Our experimental results showed that NAC reversed the effects of Rh4 on HT29 and HCT116 cells (Figures 2(a) and 2(b)). Furthermore, previous studies have shown that a steamed American ginseng root extract induced ROS generation, in addition to cell death, in CRC cells [32]. To determine whether Rh4 can also induce ROS production, we measured ROS concentrations in HT29 and HCT116 cells. The DCFH-DA assay results revealed that Rh4 increased the concentrations of intracellular ROS in a concentration-dependent manner, while Fer-1, a ferroptosis inhibitor, did not significantly reduce ROS concentrations (Figures 3(a) and 3(b)). These results showed that Rh4 triggered ROS generation and indicated that Rh4-induced ROS production is upstream of Fer-1, which means Rh4-induced ROS production is upstream of ferroptosis. NAC has been shown to reverse the ROS concentration increase in Rh4-induced CRC cells and thus reverse the inhibitory effect of Rh4 on CRC cells [24]. Therefore, the specific action mechanism of Rh4 on CRC cells after the action of NAC will not be repeated in this study. To further elucidate the anticancer mechanism of Rh4, we examined the effects of Rh4 on ferroptosis-related indicators. Rh4 could significantly induce the cellular accumulation of iron, lipid ROS, and MDA and reduce the concentration of GSH in HT29 and HCT116 cells after 48 hours of culture, the effects of which were enhanced with increasing concentrations of Rh4 (Figures 3(c)–3(f)). In addition, the increased concentrations of intracellular iron, lipid ROS, and MDA induced by Rh4 were significantly reversed by Fer-1 pretreatment. Furthermore, changes in GSH concentrations were also reversed.

Similarly, to determine whether Rh4 induces ferroptosis, we analyzed protein expression levels in cultured cells in vitro. Western blotting showed that with increasing Rh4 concentrations, the expression levels of the ferroptosis-related proteins KEAP1, NCOA4, and DMT1/SLC11A2 increased significantly. In contrast, the expression levels of NRF2, FTH1, xCT/SLC7A11, and GPX4 decreased significantly (Figures 3(g)–3(i)). Furthermore, the expression of Rh4-induced proteins was reversed by Fer-1 pretreatment. These results suggest that Fer-1 attenuates Rh4-induced ferroptosis in HT29 and HCT116 cells. Therefore, Rh4 can induce ferroptosis and inhibit CRC cell proliferation, and this process is positively correlated with intracellular ROS concentrations.

### 3.4. Ginsenoside Rh4 Induces Ferroptosis by Activating Autophagy in CRC Cells In Vitro

Investigation above experiments showed that 3-MA and Fer-1 had similar effects in inhibiting the effects of Rh4 on HT29 and HCT116 cells (Figures 2(a) and 2(b)). If 3-MA and Fer-1 acted independently, their combined effect would have boosted cell viability by more than 100%. Therefore, we hypothesized that these factors might have different targets for suppressing the same mode of death. It has been established that certain drugs can induce ferroptosis in tumor cells by activating autophagy [42]. To determine whether Rh4 can also induce ferroptosis in CRC cells by activating autophagy, we pretreated HT29 and HCT116 cells with 3-MA and then treated the cells with Rh4. Finally, we measured ferroptosis-related indicators in the cells. The results showed that the increased concentrations of intracellular iron, lipid ROS, and MDA induced by Rh4 were significantly inhibited by 3-MA pretreatment (Figures 4(b)–4(d)). Furthermore, changes in GSH concentrations were also reversed (Figure 4(a)). This finding is consistent with our hypothesis. To further determine autophagy inhibition of Rh4-induced ferroptosis in CRC, we analyzed protein expression levels in cells that were pretreated with 3-MA and then treated with Rh4. Rh4 could significantly affect the expression levels of ferroptosis-related proteins. After 3-MA pretreatment, the effect of Rh4 on the expression levels of these proteins was significantly reversed (Figures 4(e)–4(g)). These findings suggest that autophagy inhibitors can reverse Rh4-induced ferroptosis in CRC cells. Therefore, Rh4-induced ferroptosis in CRC cells is achieved by activating the autophagy pathway.

### 3.5. Ginsenoside Rh4 Promotes the Activation of p53 Signaling Pathway and Ubiquitin-Mediated Proteolysis in CRC In Vivo

To explore the mechanism of Rh4's antitumor effect in vivo, transcriptome sequencing was performed on HT29 xenograft tumor tissue. According to transcriptome sequencing results, we conducted differential analysis and found that about 3.82% (995/26031) of gene expressions were changed (up- or downregulated) after Rh4 treatment compared with control treatment (Figures 5(a) and 5(b)). The results were analyzed by GO and KEGG pathway enrichment. We found that p53 signaling pathway and ubiquitin-mediated proteolysis in HT29 xenograft tumor tissue were significantly upregulated and activated after Rh4 treatment (Figures 5(c) and 5(d)). These results suggest that Rh4 can activate the P53 signaling pathway of HT29 cells to play an antitumor role, even if HT29 cells have p53R273H mutation. At the same time, there is a close relationship between ubiquitin-mediated proteolysis and autophagy [43], and p62 and autolysosome themselves participate in the ubiquitination degradation of proteins. This suggests that Rh4 can activate autophagy in HT29 cells. These results suggest that the anti-CRC effect of Rh4 in vivo is closely related to the upregulation of p53 signaling pathway and the activation of autophagy.

### 3.6. Ginsenoside Rh4 Inhibits CRC by Activating Autophagy and Inducing Ferroptosis In Vivo

To evaluate whether Rh4 can inhibit CRC growth through ferroptosis in vivo, we analyzed xenograft tumor tissue samples from mice. In HT29 and HCT116 cell xenograft tumor tissues, the concentrations of ROS, iron, and MDA in the Rh4-treated group were higher than those in the control group (Figures 6(a), 6(c), and 6(d)), while the concentration of GSH was decreased (Figure 6(b)), which was consistent with the results of the in vitro experiments. To determine whether Rh4 activates autophagy in vivo and whether autophagy and ferroptosis both occur, we performed immunohistochemical staining analysis of key protein markers of autophagy and ferroptosis. In HT29 and HCT116 cell xenograft tumor tissues, the immunohistochemical results showed that the expression levels of the autophagy marker proteins p53 and Beclin1 were increased in the Rh4-treated group compared with the control group, while the expression levels of p62 decreased, indicating that the autophagy level in the Rh4-treated group increased compared with the control group. Furthermore, compared with those in the control group, the expression levels of the ferroptosis marker proteins xCT/SLC7A11 and GPX4 were decreased in the Rh4-treated group, indicating that the ferroptosis level was increased by Rh4 treatment (Figure 6(e)). To further confirm the increased level of autophagy in tumor tissues in the Rh4-treated group, we extracted the proteins from HT29 and HCT116 cell xenograft tumor tissues for analysis. Western blot analysis of xenograft tumor tissue indicated that p53, Beclin1, Atg7, and LC3B protein expression levels were increased compared to the control, while the p62 protein expression level was decreased (Figures 6(f)–6(h)). Similarly, ferroptosis-related proteins were analyzed. Western blot analysis of xenograft tumor tissues showed that the expression levels of the proteins KEAP1, NCOA4, and DMT1/SLC11A2, which promote ferroptosis, increased, while the expression levels of NRF2, FTH1, xCT/SLC7A11, and GPX4, which inhibit ferroptosis, decreased significantly (Figures 6(i)–6(k)). These results strongly suggest that autophagy and ferroptosis both occur during Rh4-mediated inhibition of tumor growth in vivo.

## 4. Discussion

The ginsenosides represented by Rh4 are the main bioactive constituents of steamed and heat-processed American ginseng, *Panax ginseng*, and *Panax notoginseng* extracts [25, 44]. Rh4 has previously been reported to inhibit the proliferation of various cancer cells, including esophageal cancer, breast cancer, and CRC, by inducing apoptosis and autophagy [23, 24, 45]. However, the potential of Rh4 to inhibit CRC cells and the anticancer mechanism have not been fully elucidated.

This study showed that Rh4 had high anti-CRC activity, few toxicities, and few side effects. Second, we found that Rh4 could activate autophagy and induce ferroptosis in CRC cells. Finally, we confirmed that the induction of ferroptosis was closely related to the activation of autophagy, the increase in intracellular ROS concentrations, and the activation of the p53 signaling pathway.

Rh4 inhibited the proliferation of CRC cell lines HT29 and HCT116 in a time- and dose-dependent manner in vitro. In a xenograft nude mouse model, Rh4 significantly suppressed tumor growth, and the body weights of Rh4-treated mice were slightly higher than those in the control group, without significant cardiohepatic and renal toxicity. Therefore, Rh4 has high anti-CRC activity and few toxicities and side effects.

Previous studies have reported that Rh4 can increase intracellular ROS concentrations in CRC cells and induce autophagic death, but the process of autophagic death has not been further analyzed [24]. Autophagy is a crucial regulator of cellular fate, protecting cell survival and increasing death [46]. Autophagy is an early stage defensive mechanism that can protect tumor cells after being exposed to insulting conditions while overactivity of autophagy can lead to cell death. Autophagy has a twofold effect on cancer cell survival [47,48]. Our experimental data showed that autophagy inhibitors could reverse the inhibitory effect of Rh4 on CRC cells, suggesting that Rh4-induced autophagy promoted death in CRC cells. Oxidative stress has been shown to induce or mediate p53 signaling pathway activation, which regulates autophagy [49, 50]. ROS are important indicators of oxidative stress. ROS act as upstream signals that trigger p53 signaling pathway activation [51], and activation of the p53 signaling pathway in CRC cells upregulates Beclin1 expression levels [52]. Mechanistically, Beclin1 is a crucial protein associated with autophagy initiation, which, together with PIK3C3 and PIK3R4, forms a Class III PI3K protein complex and ultimately regulates the formation and maturation of autophagosomes [53–55]. Atg7 and LC3B are markers of autophagosome formation [56, 57]. LC3B is involved in the recruitment of p62 to autophagosomes [58], and p62 is eventually degraded, decreasing the protein level of p62 [59]. In this study, we also demonstrated that Rh4 could upregulate the expression level of autophagy-related proteins, the effect of which was inhibited by the autophagy inhibitor 3-MA. Furthermore, the results showed that Rh4-induced CRC inhibition could also be blocked by NAC, and NAC may scavenge Rh4-induced ROS and reverse the inhibitory effect of Rh4 on CRC cells, which had been confirmed in a previous study [24].

In addition, unlike previous reports, we showed for the first time that Rh4 could induce ferroptosis in CRC cells. Ferroptosis, which is a new regulated form of programmed cell death, is different from apoptosis [60], necrosis [26], and pyroptosis [61]. As a novel form of iron-dependent cell death, ferroptosis is mainly induced by excessive iron and lipid peroxides, including lipid ROS and MDA. However, the specific downstream effector proteins (e.g., pore-forming proteins) and the precise mechanisms remain unclear. This death process is characterized by increased intracellular ROS, iron, and lipid ROS concentrations. Intriguingly, ferroptosis could be inhibited by antioxidant agents and iron chelation but not by inhibitors of apoptosis, necrosis, or pyroptosis [62]. MDA is an important indicator of lipid peroxidation, and GSH can inhibit lipid peroxidation [63, 64]. Lipid peroxidation results in large amounts of lipid ROS production, which ultimately leads to ferroptosis in cells. Our results showed that Rh4 could significantly increase intracellular ROS, iron, lipid ROS, and MDA levels in a concentration-dependent manner while also decreasing GSH concentrations. Notably, apoptosis, necrosis, and pyroptosis inhibitors did not affect Rh4-induced cell death in HT29 cells. However, apoptosis inhibitors reversed the inhibitory effect of Rh4 on HCT116 cells to a certain extent. This may be due to the mutation of p53R273H in HT29 cells, while HCT116 is wild type.

Nuclear factor E2-related factor 2 (NRF2) has been identified as a significant regulator of the transcription of various antioxidant genes and many other cellular protective genes [65]. After binding to KEAP1, NRF2 can be degraded through the E3 ubiquitin ligase pathway, and p62 can bind to KEAP1 to prevent NRF2 from binding to KEAP1 and being degraded. During autophagy, p62 is degraded, leading to the downregulation of NRF2 expression and decreased antioxidant levels in cells [66]. The decrease in cellular antioxidant levels leads to increased NCOA4 expression levels, which promote the degradation of FTH1 and the expression of DMT1 [67, 68]. The degradation of FTH1 leads to iron release, while DMT1 increases iron absorption, leading to iron overload in cells [69, 70]. Excess iron produces ROS through the Fenton reaction [71]. ROS further react with intracellular lipids to produce lipid ROS and MDA [72] and eventually lead to ferroptosis. On the other hand, the expression level of xCT and the activity of system Xc(−) are regulated by NRF2 [73]. A decrease in NRF2 affects the activity of system Xc(−), depletes GSH, and ultimately leads to decreased GPX4 activity. The decreased function of GPX4 affects lipid peroxidation and can result in the induction of ferroptosis [74]. After p53R273H mutation, NRF2's activation effect on system Xc(−) was weakened or even lost [75]. Therefore, both in vitro and in vitro experiments showed that after Rh4 treatment, the change of xCT/SLC7A11 in HT29 was weaker than that in HCT116. However, this did not significantly affect the effect of Rh4-induced ferroptosis in HT29 cells.

Furthermore, we found that autophagy and ferroptosis inhibitors were equally effective in reversing Rh4-mediated inhibition of CRC cell viability. Autophagy activation has been shown to induce ferroptosis in cancer cells, inhibiting cell proliferation [42, 76]. Therefore, we examined whether autophagy inhibitor preconditioning affected ferroptosis in Rh4-induced CRC cells. We examined ferroptosis markers, and the results showed that pretreatment with the autophagy inhibitor 3-MA could reverse Rh4-induced ferroptosis in CRC cells. These results suggest that Rh4-induced ferroptosis in CRC cells was mediated by the activation of autophagy. In other words, this demonstrates that Rh4 is primarily responsible for ferroptosis in CRC cells by activating autophagy, rather than directly mediating ferroptosis by activating p53. Activation of p53 signaling pathway is upstream of autophagy, and ferroptosis is downstream of autophagy.

Finally, we confirmed that Rh4 could activate autophagy and induce ferroptosis in CRC cells in vivo by transcriptome sequencing and measuring the related indicators of autophagy and ferroptosis in xenograft tumor tissues, and the results further confirmed the accuracy and reliability of the in vitro results. Therefore, we confirmed that Rh4 activated autophagy and induced ferroptosis in CRC cells, ultimately leading to tumor cell death.

The mechanism by which Rh4 inhibits proliferation and induces ferroptosis by activating autophagy in CRC cells is illustrated in Figure 7. In conclusion, autophagy activation by ROS/p53 signaling pathway upregulation is associated with Rh4-induced ferroptosis in CRC cells.

## 5. Conclusions

We found that Rh4 could induce ferroptosis in CRC cells with high anticancer efficacy and few toxicities and side effects. Ferroptosis was positively regulated by autophagy activation and was associated with increased intracellular ROS concentrations and upregulation of the p53 signaling pathway. These findings provide an alternative strategy for treating CRC and elucidate the potential anticancer mechanism of Rh4.

## Figures and Tables

**Figure 1:** Rh4 significantly inhibited the proliferation of CRC cells in vivo and in vitro. (a) The chemical structure of Rh4. (b)–(e) The viability of CRC (HT29, HCT116, DLD1, and RKO in that order) cells treated with different concentrations of Rh4 in medium for 24, 48, and 72 hours. (f), (g) Giemsa-stained colonies were observed under an inverted microscope and quantified. HT29 and HCT116 human CRC xenograft mouse models were treated with solvent or Rh4 (40 mg/kg/d). (h) Body weight was measured every 3 days (*n* = 10). (i) HE staining of heart, liver, and kidney tissues. Scale bars = 100 *μ*m. (j) Tumor size was measured every 3 days (*n* = 10). (k) Representative image of HT29 and HCT116 xenograft tumor tissues from the control (solvent) and Rh4-treated groups. Scale bars = 1 cm. (l) Xenograft tumor tissue weight after 21 days of treatment (n = 10). The data are presented as the means ± SD of triplicate experiments. (b)–(e) ^*∗∗∗*^*p* < 0.001 compared with the control group (0 *μ*M Rh4); ##*p* < 0.01, ###*p* < 0.001 compared with the 24-hour group. (g), (h), (j), (l) ^*∗∗∗*^*p* < 0.001 compared with the control group.

**Figure 2:** Rh4 activates autophagy in human CRC cell lines. (a), (b) The viability of HT29 and HCT116 cells. HT29 and HCT116 cells were pretreated with 2 mM NAC (ROS scavenger), 2 mM 3-MA (autophagy inhibitor), 2 *μ*M Fer-1 (ferroptosis inhibitor), 60 *μ*M Z-VAD (apoptosis inhibitor), 40 *μ*M Nec-1 (necrosis inhibitor), or 20 *μ*M VX-765 (pyroptosis inhibitor) for 4 hours and then incubated with 200 *μ*M Rh4 for 48 hours. (c) Effects of different concentrations of Rh4 or pretreatment with autophagy or ferroptosis before incubation with Rh4-containing medium on cell growth and morphology. Scale bars = 200 *μ*m. (d), (e) and (f) Cells were treated with Rh4-containing medium or pretreated with autophagy inhibitors, and then Rh4-containing medium was added and incubated for 48 hours. The expression levels of autophagy-related proteins were determined by Western blotting. Values are presented as the means ± SD; *n* = 3; ^ns^^*∗*^*P* > 0.05, ^*∗*^*P* < 0.05, ^*∗∗*^*P* < 0.01, ^*∗∗∗*^*P* < 0.001 compared with the control group (0 *μ*M Rh4); ^ns#^*P* > 0.05, ^##^*P* < 0.01, ^###^*P* < 0.001 compared with the 200 *μ*M Rh4 group.

**Figure 3:** Rh4 induces ferroptosis in HT29 and HCT116 cells. (a), (b) ROS concentrations were analyzed by flow cytometry after HT29 and HCT116 cells were exposed to different concentrations of Rh4 in medium with or without 1 *μ*M Fer-1 pretreatment for 48 hours; the cells were stained with DCFH-DA. (c) The relative concentration of GSH in HT29 and HCT116 cells exposed to different concentrations of Rh4 in medium with or without 1 *μ*M Fer-1 pretreatment for 48 hours. (d) Concentrations of iron in HT29 and HCT116 cells exposed to different concentrations of Rh4 in medium with or without 1 *μ*M Fer-1 pretreatment for 48 hours. (e) The relative concentrations of lipid ROS in HT29 and HCT116 cells exposed to different concentrations of Rh4 in medium with or without 1 *μ*M Fer-1 pretreatment for 48 hours. (f) Concentrations of MDA in HT29 and HCT116 cells exposed to different concentrations of Rh4 in medium with or without 1 *μ*M Fer-1 pretreatment for 48 hours. (g) Representative Western blot images of ferroptosis-related protein expression in HT29 and HCT116 cells exposed to different concentrations of Rh4 in medium with or without 1 *μ*M Fer-1 pretreatment for 48 hours. (h), (i) Relative expression levels of proteins involved in the ferroptosis pathway in HT29 and HCT116 cells exposed to different concentrations of Rh4 in medium with or without 1 *μ*M Fer-1 pretreatment for 48 hours. ns^*∗*^*p* > 0.05, ^*∗*^*p* < 0.05, ^*∗∗*^*p* < 0.01, ^*∗∗∗*^*p* < 0.001: statistically significant compared with the control group (0 *μ*M Rh4); ^##^*P* < 0.01, ^###^*P* < 0.001: statistically significant compared with the 200 *μ*M Rh4 group.

**Figure 4:** The inhibitory effect of the autophagy inhibitor 3-MA on ferroptosis induced by Rh4 in CRC cells. (a) The relative concentrations of GSH in HT29 and HCT116 cells exposed to Rh4-containing medium for 48 hours with or without 2 mM 3-MA pretreatment for 4 hours. (b) The iron concentrations in HT29 and HCT116 cells exposed to Rh4-containing medium for 48 hours with or without 2 mM 3-MA pretreatment for 4 hours. (c) The relative concentrations of lipid ROS in HT29 and HCT116 cells exposed to Rh4-containing medium for 48 hours with or without 2 mM 3-MA pretreatment for 4 hours. (d) The concentrations of MDA in HT29 and HCT116 cells exposed to Rh4-containing medium for 48 hours with or without 2 mM 3-MA pretreatment for 4 hours. (e) Representative Western blot images of ferroptosis-related protein expression in HT29 and HCT116 cells exposed to Rh4-containing medium for 48 hours with or without 2 mM 3-MA pretreatment for 4 hours. (f), (g) Relative expression levels of proteins involved in the ferroptosis pathway in HT29 and HCT116 cells exposed to Rh4-containing medium for 48 hours with or without 2 mM 3-MA pretreatment for 4 hours. ^*∗∗*^*P* < 0.01, ^*∗∗∗*^*P* < 0.001: statistically significant compared with the control group (0 *μ*M Rh4); ^##^*P* < 0.01, ^###^*P* < 0.001: statistically significant compared with the 200 *μ*M Rh4 group.

**Figure 5:** Rh4 promotes the activation of p53 signaling pathway and ubiquitin-mediated proteolysis in HT29 xenograft tumor tissue. (a) Heatmap showing the cluster of differential in Rh4 treatment and tumor control group. Up- and downregulation are represented in red and green, respectively. (b) The volcano plot of differential expression signals in Rh4 treatment and tumor control group. In the enrichment analysis of GO and KEGG pathways, the expression of Rh4 treatment group was more upregulated than that of tumor control group. (c) The bubble map of GO enrichment analyses of differential expressions in HT29 xenograft tumor tissue. The GeneRatio represents the degree of enrichment. The node size shows the number of selected genes, and the color scale represents the padj. (d) The bubble map of KEGG pathway enrichment analyses of differential expressions in HT29 xenograft tumor tissue. The GeneRatio represents the degree of enrichment. The node size shows the number of selected genes, and the color scale represents the padj. *n* = 3.

**Figure 6:** Rh4 can activate autophagy and induce ferroptosis in human CRC cells in vivo. Mice were treated with or without the Rh4. (a) Relative ROS concentrations in HT29 and HCT116 cell xenograft tumor tissues. (b) Relative GSH concentrations in HT29 and HCT116 cell xenograft tumor tissues. (c) Iron concentrations in HT29 and HCT116 cell xenograft tumor tissues. (d) MDA concentrations in HT29 and HCT116 cell xenograft tumor tissues. (e) Immunohistochemical staining was performed to analyze the expression levels of autophagy- and ferroptosis-related proteins in HT29 and HCT116 cell xenograft tumor tissues. Scale bars = 100 *μ*m. (f) Western blotting was performed to analyze the expression level of autophagy-related proteins in HT29 and HCT116 cell xenograft tumor tissues. (g), (h) Relative expression levels of autophagy-related proteins in HT29 and HCT116 cell xenograft tumor tissues. (i) Western blotting was performed to analyze ferroptosis-related protein expression levels in HT29 and HCT116 cell xenograft tumor tissues. (j), (k) Relative expression levels of ferroptosis-related proteins in HT29 and HCT116 cell xenograft tumor tissues. ^*∗∗*^*P* < 0.01, ^*∗∗∗*^*P* < 0.001: statistically significant compared with the control group (solvent).

**Figure 7:** Schematic illustration of the potential underlying mechanism responsible for Rh4-induced ferroptosis.

## Data Availability

The datasets used and/or analyzed during the current study are available from the corresponding author on reasonable request. Original datasets for transcriptome sequencing can be obtained by accessing the NCBI Trace Archive or NCBI Sequence Read Archive (URL: https://www.ncbi.nlm.nih.gov/Traces/study/?acc=PRJNA826695).
